RETRACTED

# A Plain Bayesian Algorithm-Based Method for Predicting the Mental Health Status and Biomedical Diagnosis of University Students

**DOI:** 10.1155/2022/2617488

**Published:** 2022-08-28

**Authors:** Jiao Wang

**Affiliations:** Center for Ideological and Political Education & Guidance Center for Student Psychological Development, Northeast Normal University, Changchun 130024, China

## Abstract

The purpose of this study was to assess e-learning during Corona epidemic regarding advantages, limitations, and their recommendations for managing learning during the epidemic. Based on a case study, this study used qualitative research. Sixteen students from King Saud University's College of Education were invited to take part. These students receive their online lectures via the “Zoom” application. A 20-minute WhatsApp one-on-one semiorganized interview was likewise utilized. To guarantee the reliability, iCloud was utilized to record gatherings and meetings for direct record (adaptability, constancy, confirmability, and validity). Results were presented in three themes: advantages of employing distance education, limitations of usages, and recommendations for improvements. Analyzing the feedbacks collected from students by the four interviewers, important characteristics of distance education emerged. They were student-centered learning, which included: comfortable, self-directed learning, asynchronous learning, and flexibility. The most common limitations associated with distance education, in general, included inefficiency, that is, lack of student feedback, and lack of attentiveness. As for recommendations for improvements the most obvious characteristics that became evident in students' responses were teaching and assessment and quality enhancement.

## 1. Introduction

Since the beginning of 2020, the world has witnessed exceptional circumstances associated with the prevalence of the new Corona virus or Covid-19 [1]. Educational institutions have been affected by these decisions, and it is no longer possible to continue the educational process in its traditional form, and millions of students and their teachers at all educational stages have been kept in their homes. The form of the spread of this virus or the Corona epidemic is a major crisis that all countries of the world faced without exception, and the countries of the world rushed to search for alternative methods to prevent the educational process from stopping, and not all countries were at the same level in dealing with this emergency situation. Different experiences emerged to deal with this emergency, and this was followed by the emergence. The term emergency remote education is along with the term e-learning, and UN institutions such as UNESCO [2] and other institutions have intervened to follow this emergency matter and provide a helping hand to various countries of the world, given that this epidemic has formed a common denominator for the suffering of millions of people worldwide, and part of that suffering is due. To the fears associated with the spread of the epidemic and the number of daily deaths, and the denial of the practice of normal humanitarian activity.

RETRACTED

### 1.1. Saudi Arabia Experiences in Applying E-Learning during Corona Epidemic

The Kingdom of Saudi Arabia has a rich experience in managing crises facing the educational process. This appeared at the southern border. In 2016, a distance education program was signed, in cooperation between the Ministry of Education and the Education Development Company, and the Minister of Education stated at the time that providing this quality service in the educational field is a duty to enable students to continue their learning under any circumstances and that the Education Development Company has prepared for this program and has the capabilities to fully implement it to help provide education and service at this time, especially for those affected by crises, indicating that the Ministry of Education provided educational alternatives in the southern border and benefited from developing electronic programs and broadcasting some programs through TV channels prepared for this purpose, and he confirmed the Ministry's readiness to provide assistance at any time in all circumstances [3, 4].

As for the management of the crisis that resulted from the Corona epidemic, the Saudi Ministry of Education announced the closure of various educational institutions since the eighth of March in accordance with the Noble Decree No. (42874), and a specialized committee was formed in the Ministry of Education to follow up the developments of the spread of the Corona epidemic, and the Ministry took the initiative to define a variety of packages.

As per the Saudi Ministry of Education, e-learning stages for public and private schooling have been actuated, notwithstanding the accompanying critical measures.

The virtual school building was finished in multi week, during which the school's central command and satellite telecom were outfitted, 20 savvy sheets were provided and introduced, and the school personnel was prepared to photo educational clasps.

With the assistance of 276 educators and 73 bosses, everyday examples were ready to make sense of the educational program. 3368 examples were made sense of, adding up to 1684 hours of educating time.

In addition to the curriculum review lessons, 123 teachers and 73 supervisors participated. 1107 lessons were reviewed, totaling 554 hours of teaching time.

RETRACTED

The Ministry carried out distance education involving the techniques for synchronous collaboration and nonconcurrent communication as follows.

Concurrent connection was accomplished through the virtual school application, which incorporated the bound together education framework, the eye entryway, the door representing things to come, and the virtual kindergarten application. Nonconcurrent connection was utilized by means of Ain satellite stations and Lessons Ain stations on YouTube. The past stations and stages gave numerous choices to male and female students to proceed with education and advancing from a distance, by means of the Internet or through satellite stations, for the people who do not approach the Internet, and these stations saw a ton of collaborations among male and female students and contributed extraordinarily to the fruitful continuation of the educational cycle. Following is a short outline of these channels.

Future Gate is a coordinated e-learning stage for students, all things considered. It has received over 20 million visits, and its services have benefited over 700,000 students.

Ain Satellite Channels are an assortment of 20 satellite stations that cover every single educational level. The channels are functional 24 hours a day, seven days a week.

Ain Channels on YouTube: These are live YouTube channels with more than 60 million perspectives.

Ain (National Education Portal): The gateway offers advanced content that incorporates more than 45,000 virtual educational materials and north of 2000 computerized books.

Virtual Kindergarten is a thorough educational framework for the youth stage.

The framework contains advanced educational illustrations and exercises in an intelligent educational climate between the educator and the understudy. The Ain stage gives day-to-day clarifications of the educational plans for every educational stage, and the Kingdom's choice to enact the “Board” framework came following the spread of the Corona infection, and the framework gives many advantages to instructors, including the following:

  Keeping track of student attendance and absences.
  Students can be given assignments, tests, and courses.
  Create virtual lessons.
  Make educational ways for a select gathering of students.
  Answer understudy requests sent through educator rooms.

The brought-together education framework site has become one of the most noticeable arrangements that anyone could hope to find for distance education in the Kingdom of Saudi Arabia to speak with students, and it remembers all administrations connected with education for Saudi Arabia for all male and female students. This short show of the Kingdom of Saudi Arabia's experience shows that there are numerous choices accessible to male and female students in the Kingdom to follow the educational cycle and to furnish distance education with various options through the Internet or satellite stations, as well as the Ministry of Education's nearby drive to go to the vital lengths and not stop educational administrations for all degrees of education. The Saudi experience concurred with its partner in the United Arab Emirates, as the UAE has broad experience and mastery in the field of involving innovation in education, and this experience varied from past encounters, which saw a stoppage in the use of distance education methods or a more prominent accentuation on the utilization of the Internet around here.

RETRACTED

The Saudi Ministry of Education's drive to manage the Corona plague, and the danger it postures to the educational cycle can be made sense of considering the Kingdom's past involvement with overseeing educational emergencies, as the Saudi Ministry of Education had past rich involvement with giving distance education administrations to male and female students on the Kingdom's southern lines, and the arrangement included distance education administrations. It safeguarded the understudy's principal privileges to education by placing him in direct contact with his educators through the school twinning venture. Other electronic educational options, for example, the “illustrations” educational stations and the “AAli” satellite station, were likewise enacted, with the stages of online education benefiting.

## 2. Objective

The goal of this study was to evaluate e-learning during Corona epidemic regarding advantages, limitations, and their recommendations for managing learning during the epidemic.

## 3. Method

### 3.1. Design

This study utilized qualitative case study research, in which the scientist examines a reality, contemporary limited framework or various limited frameworks over the long run by social event definite, top to bottom data and detailing case subjects and case depictions [5].

### 3.2. Participants and Procedures

Sixteen students from King Saud University's College of Education were invited to take part. These students received their online lectures via the “Zoom” application. Furthermore, a 20-minute WhatsApp one-on-one semiorganized interview was utilized [6]. To guarantee dependability, iCloud was utilized to record gatherings and meetings for direct record (transferability, dependability, confirmability, and credibility). Four interviewers; the author besides three other lecturers, conducted the interviews. The data were thematically analyzed: compiling, disassembling, reassembling, and interpretation by all the interviewers each on his own, and then the data were corroborated to ensure analytical accuracy [5].

RETRACTED

## 4. Results

### 4.1. Presentation of Findings

Results were presented in three themes: Advantages of employing distance education, limitations of usages, and recommendations for improvements.

**Theme 1 .**

*Advantages of employing distance education*. Analyzing the feedbacks collected from students by the four interviewers, an important characteristic of distance education emerged. It is student-centered learning, which includes comfortable, self-directed learning, asynchronous learning, and flexibility. For example, the majority of the students agreed with Student 18, who stated, “*It is easy and more comfortable for me now to listen to the lecture while sitting in my bedroom*, *or anywhere that I get used to and feel comfortable*” [7]. This new learning climate focused on electronic organizations has empowered college students to get individualized help along with learning plans that are more reasonable to them and separate from other students. Obviously, e-learning can empower students at higher educational levels to get their education while likewise seeking after their own objectives and keeping up with their own professions, without sticking to an inflexible timetable [8].

As for Self-directed Learning, a large portion of the understudies concurred with Student 3 who placed, “*I think Distance Education is making good students more active and self-learner*, *that is*, *it helps them in becoming engaged with growing experiences like securing data*, *arranging*, *and assessing learning exercises*.” All in all, independent students ordinarily take part more effectively in learning errands, for example, perusing web-based learning material, finishing homeroom assignments, and arranging and assessing learning achievements [9]. An independent student effectively takes part in growing experiences like data securing, arranging, and assessing learning exercises. Dynamic learning systems can help understudy investment while additionally further developing learning and execution [10, 11].

Concerning asynchronous learning, a large portion of the understudies concurred with Student 7 who set, “*One can download lectures at any time*. *It is easy for us to go back and go through the whole video for revision*.” Asynchronous learning, in other words, assists in making learning self-paced, independent, and, most importantly, student-centered [12]. Accordingly, this sort of learning is probably going to framework students' earlier information with new ideas [13], it allows for peer group discussions, and it promotes decisive reasoning and profound learning [14].

RETRACTED

As for flexibility, the majority of the students agreed with Student 18, who proposed, “*Although we are away from our university*, *and cannot attend lectures*, *however*, *distant learning during COVID 19 enables us to continue our education and have all our lectures without discontinuity*.” As such, students have more opportunity in choosing when, how, and with what content and exercises they take part in web-based learning situations [15]. This versatility requires students checking and changing their way of behaving and activities comparable to the particular learning setting (Zimmerman, 2000).

**Theme 2 .**

*Limitations of usages*. Analyzing the feedbacks collected from students by the four interviewers, students reported some Limitations of usages, concerning distance learning. The most obvious characteristic that became evident in student's responses was inefficiency, which included lack of student feedback and lack of attentiveness. Concerning lack of student feedback, the vast majority of the understudies concurred with Student 2 who set, “*the professor does not know for sure whether his students are getting the point or not*. *That is*, *he does not care much of getting students feedback*. *He only gives the lecture as if it were a chore to do*.” In other words, due to the epidemic, higher institutions in every corner of the world, including my country as well, are compelled to suspend up close and personal classes. That is, they have rushed to remote teaching and online classes, posing unprecedented challenges in terms of learning new technologies and gaining access to necessary facilities such as laboratories [16].

Concerning lack of attentiveness the majority of the understudies concurred with Student 15 who set, “*I think that type to instruction has some limitations such as lacking students attention* . *why? Students know that they will get the recordings at any time*, *so they might not listen the lecture properly*.” In other words, in a real-world classroom, a teacher easily captures students' attention and adapts lessons accordingly to maximise student interest and participation [17]. However, in distance education, students feel free to attend or not attend to the lecturer, as they think they will get the recordings at any time.

**Theme 3 .**

*Recommendations for improvements*. Analyzing the feedbacks collected from students by the four interviewers, students reported some recommendations for improvements, concerning distance learning. The most obvious characteristics that became evident in students responses were teaching and assessment and quality enhancement. Teaching and assessment included online examination. As for online examination, the majority of the understudies concurred with Student 6 who set, “*online examination helps university teachers to reach remote students*.” Another student (Student 3) proposed that “*the online examination may result in an equal level of student performance*.” Another student (Student 17) stated that “*online examination helps to boost students' results*.” As such, students favor electronic appraisals since they have more control, easy to use points of interaction, and tests that look like learning conditions and sporting exercises. When contrasted with paper tests, e-appraisal gives quick criticism, which supports the improvement of learning levels. This is consistent with the findings of [18–20].

RETRACTED

As for quality enhancement, majority of the students agreed with Student 1 who stated, “*Being out of sight of their instructors*, *will allow students to collaborate together*, *thus writing the same assignments from the same source*. *I think*, *there should be plagiarism software to check assignment*.” Some researchers blame the Internet for the increased “opportunities” for cheating [21], while others believe the increased incidence of cheating is due, at least in part, to the use of Internet [22].

## 5. Discussion

The goal of this study was to evaluate e-learning during the Corona epidemic regarding advantages, limitations, and their recommendations for managing learning during the epidemic. Results were presented in three themes: advantages of employing distance education, aimitations of usages, and recommendations for improvements. Analyzing the feedbacks collected from students by the four interviewers, important characteristics of distance education emerged. They were Student-centered learning, which included:comfortable, self-directed learning, asynchronous learning, and flexibility. This is consistent with findings, which determined that flexible learning, defined as a learner-centered approach to learning, provided students with different learning options, which in turn helps to make learning outcomes useful and exciting [23–26]. During the COVID-19 pandemic, we require enough time to extend and sustain online education.

The most common limitations associated with distance education in general included the inefficiency, that is, lack of student feedback and lack of attentiveness. In the traditional classroom, students meet each other in the space; exchange ideas, information, and knowledge; ask the professor; interact with them; and receive feedback from colleagues and teachers, while sharing ideas, knowledge, and information in real time in the virtual environment, i.e., in distance learning, is considered missing to a large extent. Concerning reported limitations, this result, in the same line, indicates it is absurd to teach students through distance learning without preparing the climate, environment, and students for this type of learning [27]. Teachers should be skilled, on one hand, and students should be prepared for this, on the other hand.

RETRACTED

With the advent of social media, students now have instant access to a wealth of information. Internet search results are also electronic, and students can easily copy and paste the information into assignments, papers, and other documents [28].

## 6. Conclusion

This paper points to assess e-learning during the Corona epidemic regarding advantages, limitations, and their recommendations for managing learning during the epidemic. Results were presented in three themes: advantages of employing distance education, limitations of usages, and recommendations for improvements. Analyzing the feedbacks collected from students by the four interviewers, important characteristics of distance education emerged. They were Student-centered learning, which included comfortable, self-directed learning, asynchronous learning, and flexibility, inefficiency, which included ack of student feedback, and lack of attentiveness, and teaching and assessment and quality enhancement. Teaching and assessment included online examination and Quality enhancement.

## Data Availability

The data used to support the findings of this study are included within the article.
